RETRACTED

# Study on Transmission Channel and Pollution Sources Region of O_3_ in Qingyuan City

**DOI:** 10.1155/2022/1837492

**Published:** 2022-09-15

**Authors:** Cuihua Li, Mai Boru, Yangbin Li, Jingman Peng, Qingxi Huang

**Affiliations:** ^1^Meteorological Bureau of Qingyuan, Qingyuan 511500, China; ^2^Institute of Tropical and Marine Meteorology, China Meteorological Administration, Beijing, China

## Abstract

Based on the Lagrange mixed single-particle trajectory model and NCEP global reanalysis meteorological data, the 72 h backward airflow trajectory in Qingyuan City in different seasons from 2018 to 2020 was analyzed by cluster analysis. Combined with the hourly average concentration data of O_3_, the potential source contribution factor (PSCF) analysis and concentration weighted trajectory (CWT) analysis were used to study the regional transport and possible source area of O_3_ in Qingyuan City and analyzed the relationship among O_3_ and wind speed, wind direction, NO_2_, and CO. The results showed that from 2018 to 2020, the most significant proportion of primary pollutants in Qingyuan City was ozone. The annual average concentration reached the highest value since monitoring in 2019. In 2020, the impact of epidemic prevention and control decreased. The daily average concentration change characteristics showed a single peak, with the highest concentration in the afternoon, the highest peak concentration in summer, followed by spring, and the lowest concentration in winter. There are differences in the concentration of O_3_ between different sources of airflow in Qingyuan City. The potential source contribution factor shows that the high-value covered areas are mainly in Guangzhou, Foshan, and Zhongshan, which can be considered the main potential source areas. These areas can be regarded as the main potential source areas. The concentration weight trajectory showed that external and local sources affected the O_3_ pollution in Qingyuan during the four seasons. The high ozone concentration in Qingyuan mainly appeared in the south wind direction, indicating that the high ozone concentration in Qingyuan was greatly affected by the external transmission of the southern Pearl River Delta. The correlation between ozone concentration and CO concentration is poor, and the effect on ozone concentration is less than that of NO_2_.

## 1. Introduction

The ozone (O_3_) near surface is a secondary pollutant generated by complex photochemical stress such as VOCs and NOx, hurting human health, crop growth, and yield. In the meantime, O_3_, as a greenhouse gas, also impacts global climate change. In recent years, the PM_2.5_ pollution in China improved significantly, but the O_3_ pollution has risen in most cities, and the problem is increasingly prominent. O_3_ has a relatively long service life and is easy to form regional transmission. Therefore, the local O_3_ concentration is affected by the photochemical reaction of locally discharged precursors and the news of O_3_ or precursors generated in the field. Identifying the sources of O_3_ is an essential premise for formulating accurate and effective control measures.

RETRACTED

In recent years, many cities and regions in China have begun to study the pollution of O_3_ (e.g., [1, 2], Guangdong is one of the earliest O_3_ research areas in China. Relevant studies mainly focus on the various characteristics of O_3_ concentration [3], the relationship between O_3_ and precursors (VOCs, NOx, and CO), and meteorological conditions [4–6], as well as qualitative correlation analysis and model simulation on a short time scale. However, it is rare to study the variation law of O_3_ based on years of hourly observation data and the source of O_3_.

Qingyuan is located north of Guangdong, adjacent to the Guangdong-Hong Kong-Macao Greater Bay Area, and only 60 kilometers from Guangzhou. The problem of O_3_ pollution in this area has been prominent in recent years. Qingyuan has carried out relatively standardized O_3_ concentration monitoring since October 2013, after the promulgation of the new ambient air quality standard in 2012. Based on hourly ozone concentration monitoring data and NCEP reanalysis meteorological data of two ambient air quality national control stations in Qingyuan from 2018 to 2020, the transmission path, transmission process, and distribution characteristics of the potential source region of pollutants in Qingyuan City in four seasons are analyzed step by step by using the split backward trajectory model and PSCF and CWT methods. Quantitatively determining the transmission contribution among different regions, provinces, and cities can provide a scientific basis for the prevention and control of air pollution in Qingyuan City and be of great significance for the coordinated prevention and control of air pollution between adjacent cities.

## 2. Data and Methods

### 2.1. Data

The hourly mass concentration data of O_3_ used in this study are selected from two national environmental monitoring points in Qingyuan City from 2018 to 2020. The airflow trajectory data are the data of the global data assimilation system (GDAS), provided by NCEP. The elements related to the meteorology of the data include air pressure, temperature, relative humidity, and vertical and horizontal wind speed. The vertical direction is divided into 23 layers, and the spatial resolution is 0.5° × 0.5°, recorded once every 6 hours, respectively, at 00 : 00, 06 : 00, 12 : 00, and 18 : 00 (UTC).

RETRACTED

The HYSPLIT model is an integrated model system jointly developed by the Air Resources Laboratory of the National Oceanic and Atmospheric Administration (NOAA) and the Bureau of Meteorology Australia [7, 8]. It is a diffusion model mixed by Euler and Lagrangian, which has a relatively complete process of transportation, diffusion, and sedimentation. At present, it has been widely used in the analysis of transmission paths and sources of air pollutants [4, 9].

In this paper, we took the Qingyuan area (23° 72′N, 113° 09′E) as the simulated site, and the starting height of the trajectory is 500 m from the ground. Using the GDAS meteorological data of NCEP calculated the 72 h backward airflow trajectory reaching Qingyuan City at 00 : 00, 06 : 00, 12 : 00, and 18 : 00 (Beijing time) from January 2018 to February 2021. The 72 h backward trajectory of airflow can well reflect the characteristics of cross-regional transmission of pollutants and cover the life cycle of secondary pollutants [10, 11].

### 2.2. Cluster Analysis

Cluster analysis is a multivariate statistical technique to classify samples by mathematical methods according to their similar characteristics. Backward trajectory clustering is to regroup and cluster a large number of airflow trajectories according to the moving speed, spatial similarity, and direction of air mass trajectories, so as to obtain the airflow in the dominant direction, potential sources of pollutants, and specific pollutant transport channels. TrajStat software has two clustering methods: Euclidean distance and angular distance. This paper mainly studies the direction of the airflow trajectory reaching the receiving point, so the latter is adopted in this paper. Grid the study area to 0.25° × 0.25° horizontal grid, cluster PSCF and CWT analyses are carried out in the Qingyuan area by TrajStat software [12], and different transmission airflow types and potential source regions in four seasons are obtained.

### 2.3. Potential Source Contribution Analysis

PCSF (potential source contribution function) is also called the residence time analysis method [13]. It is based on the backward trajectory calculation of air mass to identify the pollutant source area [14, 15], which was applied to TrajStat software. PCSF value is defined as the ratio of the number of contaminated tracks (*m*_*ij*_) passing through the grid *ij* to the number of all tracks (*N*_*ij*_) passing through the grid [16].

(1) $$\begin{array}{c} {\text{PSCF}}_{ij}=\frac{m_{ij}}{n_{ij}}. \end{array}$$

In this paper, the maximum daily average secondary concentration limit 8-hour 160 *μ*g·m^−3^ of O_3_ is used as the judgment criterion for whether the trajectory is polluted or not. When the pollutant concentration corresponding to the air mass trajectory passing through a grid reaches Qingyuan and exceeds the secondary standard limit, the trajectory is a pollution trajectory. Otherwise, it is a cleaning trajectory. The high-value grid area of PCSF is considered the potential source region of O_3_ in Qingyuan City. PSCF is a conditional probability. When the overall residence time of the trajectory of some remote grids is small, the result is very uncertain. Therefore, *W*_*ij*_ (weight factor) [17] is introduced to reduce it. When *N*_*ij*_ in a grid is less than three times the average trajectory endpoints in each grid in the selected study area [18], *W*_*ij*_ calculation should be used to reduce the uncertainty of PCSF. The calculation formula is

(2) $$\begin{array}{c} \text{WPSCF}=W_{ij}\cdot \text{PSCF}, \end{array}$$

and *W*_*ij*_ is defined as follows:

(3) $$\begin{array}{c} W_{{}_{ij}}=\left\{\begin{array}{c} 1.0080\leq n_{ij}\\ 0.7020<n_{ij}\leq 80\\ 0.4210<n_{ij}\leq 20\\ 0.05<n_{ij}\leq 10 \end{array}\right\}. \end{array}$$

RETRACTED

### 2.4. Concentration Weighted Trajectory (CWT) Analysis

The PCSF method has limitations in reflecting the grid pollution trajectory. When the pollutant concentration is higher than the set standard, the weight of the grid unit can be the same, which cannot sufficiently reflect the pollution degree of the pollution trajectory. Therefore, the weighted concentration of trajectory is calculated by concentration weighted trajectory analysis (CWT) to compensate for this deficiency. Quantitatively give the average weight concentration of each grid and reflect the pollution degree of different trajectories [19]. The specific methods are as follows:

(4) $$\begin{array}{c} C_{ij}=\frac{1}{\sum_{l=1}^{M}\tau_{ijl}}\sum_{l=1}^{M}C_{l}\tau_{ijl}, \end{array}$$

where *C*_*ij*_ is the average weight concentration of the cell grid (*i*, *j*), *l* is the trajectory, *M* is the total number of tracks, *C*_*l*_ is the corresponding pollutant mass concentration when the trajectory passes through the grid, and *τ*_*ijl*_ is the residence time of trajectory *L* in the grid (*i*, *j*) [20, 21]. The same weight factor *W*_*ij*_ as PCSF is adopted to reduce the uncertainty of *C*_*ij*_.

(5) $$\begin{array}{c} \text{WCWT}=C_{ij}\times W_{ij}. \end{array}$$

## 3. Results and Analysis

### 3.1. Ozone Pollution Characteristics

The most significant proportion of primary pollutants in Qingyuan (Figure 1) is ozone. From 2018 to 2020, the number of days with ozone as the primary pollutant accounted for 53.8% of the total monitoring days increased to 59.9%, showing an increasing trend year by year. The problem of ozone pollution has become increasingly prominent.

RETRACTED

Figure 2 shows the daily variation characteristics of ozone in Qingyuan City from 2018 to 2020. The daily average concentration range is 0.5–160 *μ*g·m^−3^, and the concentration value fluctuates wildly. The average ozone concentration in 2018 was 139 *μ*g·m^−3^, and the monitoring of ozone concentration in 2019 changed from standard to actual. Under the state transition condition, the average ozone concentration in 2019 was 152 *μ*g·m^−3^, which increased by more than 9% based on 2018, reaching the highest value since monitoring. Ozone concentrations fell to 143 *μ*g·m^−3^ in 2020 due to epidemic prevention and control.

Figure 3 shows ozone's seasonal and diurnal variation characteristics in Qingyuan City. The daily variation characteristics show a single peak type. The single peak time in different seasons is roughly the same (8 : 00–19 : 00). The highest concentration occurs at 13 : 00–16 : 00 p.m. and the lowest concentration occurs at 2 : 00–6 : 00 a.m., which is similar to the high temperature of the day, the intense sunlight, the strengthening of photochemical reactions, and the ozone precursors such as nitrogen oxides and hydrocarbons are more likely to convert into ozone. With the increase in temperature, the ozone concentration will also increase, but the attention will decrease after the sun goes down and at night. The peak concentration was the highest in summer, followed by spring, and the lowest in winter.

### 3.2. Backward Trajectory Cluster Analysis

Using the cluster analysis tool of TrajStat software, the airflow trajectory from January 2, 2018, to February 29, 2021, is classified according to its transmission speed and direction (Figure 4).

In spring, the airflow is mainly from the east direction. The southeast airflow through Zhongshan and Guangzhou cities accounted for the most significant proportion of airflow track (track 1), accounting for 38.59%, followed by the northeast airflow through Hunan Province and Shaoguan City (track 2), accounting for 31.97%. The southwest airflow through Jiangmen, Foshan, and Guangzhou (track 3) accounted for 29.44%. There is little difference in the proportion of the three airflows.

In summer, the airflow is mainly from the south direction. The south airflow through Jiangmen, Foshan, and Guangzhou (track 1) accounts for the most significant proportion of the airflow in this season, accounting for 58.79%. The southeast airflow comes from track 2 of Huizhou and Guangzhou, accounting for 26.99%. The northeast airflow comes from track 3 of Jiangxi Province, Hunan Province, and Shaoguan City, accounting for 14.22%.

RETRACTED

In autumn, the airflow is mainly from the northeast direction. The northeast airflow comes from Hubei, Jiangxi, and Shaoguan (track 1), accounting for 67.03% of the airflow this season. The southeast airflow comes from Shantou Jieyang, Shanwei, Huizhou, and Guangzhou, accounting for 24.63%. The southerly airflow comes to Jiangmen, Fushan, and Guangzhou, accounting for 8.33%.

In winter, the airflow is mainly from the northeast and southeast. The airflow comes from Shenzhen, Dongguan, and Guangzhou (track 1), accounting for 53.04%.

### 3.3. Pollution Source Analysis

#### 3.3.1. Analysis of PSCF

Cluster analysis can only distinguish the impact of O_3_ precursors brought by air masses from different regions on observation point O_3_ from the trajectory direction. It cannot further judge the geographical location of the source of O_3_ precursor. Therefore, we need to further analyze the geographical distribution of O_3_ precursor sources by using the PSCF and CWT models embedded in the TrajStat plug-in. In this paper, the maximum daily 8-hour average secondary concentration limit of O_3_ is 160 *μ*g·m^−3^ as the judgment standard of whether the trajectory is polluted or not. When the pollutant concentration corresponding to the air mass trajectory passing through a grid reaches Qingyuan and exceeds the secondary standard limit, the trajectory is a pollution trajectory. Otherwise, it is a cleaning trajectory.

The four seasons' potential source contribution factor analysis (WPSCF) of O_3_ in Qingyuan from 2018 to 2020 is shown in Figure 5. The color in the figure represents the contribution level of the potential source region. The darker the color, the greater the WPSCF value and the more significant the contribution of the grid area to the O_3_ mass concentration in Qingyuan City.

In spring, there is a potential contribution source zone of the southwest trend in Jiangmen, Foshan, and other regions (0.2 < WPSCF < 0.4).

In summer, the high value of WPSCF is in Shaoguan and Fogang.

In autumn, the WPSCF ultrahigh-value area (WPSCF > 0.6) is mainly in Guangzhou.

In winter, there are high WPSCF value areas in Zhongshan, Foshan, and Guangzhou (0.2 < WPSCF < 0.6).

We can see that the WPSCF distribution of O_3_ in Qingyuan City has seasonal characteristics, and the seasonal changes in potential contribution source areas are different.

#### 3.3.2. The Analysis of CWT

The potential source region identified by the WPSCF method can only reflect the contribution rate of the reaction potential source region, cannot reflect the specific contribution level to the target grid, and cannot distinguish the source strength [22]. Therefore, according to formulas (4) and (5), i.e., concentration weighted trajectory (CWT) analysis, the pollutant mass concentration of the potential source grid is weighted to reflect the pollution degree of the possible pollution source area (Figure 6). The darker the grid color in the figure, the greater the value, indicating that the region contributes more to the pollutant concentration in Qingyuan City.

RETRACTED

In spring, the high-value areas of WCWT (50 *μ*g·m^−3^ < WCWT < 80 *μ*g·m^−3^) in Jiangmen, Zhuhai, Foshan, Guangzhou, and Qingyuan are connected, indicating that O_3_ pollution in Qingyuan is affected by both foreign and local sources in spring.

In summer, the range of high WCWT (40 *μ*g·m^−3^ < WCWT < 60 *μ*g·m^−3^) value areas is more expansive, and the WCWT values of Yangjiang, Jiangmen, Foshan, Guangzhou, and Qingyuan are more significant, indicating that O_3_ pollution in Qingyuan in summer is also affected by foreign and local sources.

In autumn, WCWT (50 *μ*g·m^−3^ < WCWT < 80 *μ*g·m^−3^) high-value areas in Jiangmen, Zhaoqing, Foshan, Guangzhou, and Qingyuan are connected into a piece, indicating that O_3_ pollution in Qingyuan in autumn is affected by both foreign and local sources.

In winter, both sides of the Pearl River Estuary to Guangzhou and Qingyuan are high-value areas of WCWT (50 *μ*g·m^−3^ < WCWT < 80 *μ*g·m^−3^), indicating that O_3_ pollution in Qingyuan in autumn is affected by both foreign and local sources.

It can be seen that O_3_ pollution in Qingyuan in the four seasons is affected by both local and foreign sources.

### 3.4. The Relationship between O_3_ and Wind Speed and Direction

The correlation coefficients between ozone concentration and average wind speed in different spring, summer, autumn, and winter seasons in Qingyuan from 2018 to 2020 are calculated to analyze the relationship between ozone and wind.  Table 1 shows that the correlation between ozone concentration and average wind speed in different seasons of Qingyuan is relatively weak, except for the high correlation in summer (*R* = 0.29). In addition, Table 1 also calculated the correlation between ozone concentration and the days of the first wind, the second wind, and the third wind in different seasons. The correlation coefficient between ozone concentration and the days of the third wind is the highest in Qingyuan spring.

The influence of wind on the concentration of near-surface ozone and other atmospheric pollutants is reflected in the wind speed migration ability and elimination efficiency of atmospheric pollutants and the direction of pollutant transmission.  Figure 7 shows the relationship between O_3_ and wind speed and wind direction in Qingyuan City seasons. It can be seen from the figure that in Qingyuan, the high value of O_3_ in spring mainly occurs in the southwest wind direction. Summer high O_3_ mainly occurs in the south wind direction; the high-value O_3_ in autumn mainly occurs in the northeast wind direction and the southerly wind direction; winter high O_3_ mainly occurs in the south wind direction. It can be seen that the high ozone concentration in Qingyuan mainly occurs in the south wind direction, indicating that the high ozone concentration in Qingyuan is greatly affected by the external transmission of the southern Pearl River Delta.

RETRACTED

### 3.5. Correlation Analysis between Ozone Concentration and CO and NO_2_ Concentration

Since CO and NO_2_ are the main precursors of ozone, the correlation between ozone and them is analyzed in this paper. From the correlation analysis of ozone concentration and CO and NO_2_ concentration in four seasons in Qingyuan (Table 2), the correlation between ozone concentration and CO concentration is poor. The main reason is that CO is relatively inert in atmospheric chemical reactions and has less influence on ozone concentration than NO_2_.

## 4. Conclusion

1. From 2018 to 2020, the most significant proportion of primary pollutants in Qingyuan City was ozone, which showed an increasing trend yearly. In 2020, affected by epidemic prevention and control, ozone concentration decreased. The diurnal variation of ozone concentration showed a single peak type, with a single peak time (8 : 00–19 : 00). The highest concentration appeared from 13 : 00to 16 : 00 in the afternoon, and the lowest concentration appeared from 2 : 00 to 6 : 00 in the morning. The reason was that the daytime temperature was high, the sunlight was strong, and the photochemical reaction was intense.
2. The WPSCF distribution of O_3_ in Qingyuan City has seasonal characteristics, and the four season changes of potential contribution source areas are different. The WPSCF high coverage areas are mainly located in Guangzhou, Foshan, Zhongshan, and other areas considered the main potential source areas.
3. Based on the weighted concentration weighted trajectory (WCWT), it is shown that O_3_ pollution in Qingyuan during the four seasons is affected by both local and external sources
4. The high ozone concentration in Qingyuan mainly occurs in the south wind direction, indicating that the high ozone concentration in Qingyuan is greatly affected by the external transmission of the southern Pearl River Delta
5. The correlation between ozone concentration and CO concentration is poor. The main reason is that CO has relatively large inertness in atmospheric chemical reactions, which has less influence on ozone concentration than NO_2_.

RETRACTED

## Figures and Tables

**Figure 1:** Location of the Qingyuan City.

**Figure 2:** Temporal variation of ozone concentration from 2018 to 2020.

**Figure 3:** Characteristics of changes in hourly concentration of ozone matter in four seasons in 2018–2020.

**Figure 4:** Clustering of the backward trajectory of airflow in Qingyuan City from 2018 to 2020.

**Figure 5:** PSCF distribution of O_3_ in Qingyuan City in different seasons.

**Figure 6:** CWT distribution of O_3_ in Qingyuan City in different seasons.

**Figure 7:** Relationship between O_3_ and wind speed and direction in different seasons in Qingyuan City.

**Table 1:** Correlation coefficients of ozone with average wind velocity and a number of days with level 1, level 2, level 3, or above.

Season	Average wind velocity	Number of days with wind level 1	Number of days with wind level 2	Number of days with wind level 3 or above
Spring	−0.02	−0.45	0.23	0.67
Summer	0.29	0.11	−0.40	0.41
Autumn	−0.02	−0.50	−0.06	0.19
Winter	−0.18	−0.02	0.26	−0.24

**Table 2:** Correlation coefficients of ozone with CO and NO_2_.

	Spring	Summer	Autumn	Winter
CO	−0.27	0.27	−0.2	0.25
NO_2_	−0.32	0.3	0.24	0.52

## Data Availability

The data used to support the findings of this study are included within the article.
